The article "Aberrant methylation of SPARC in human lung cancers" was retracted in 2013. Reasons: misconduct by an author; duplicated data.

# Aberrant methylation of *SPARC* in human lung cancers

**DOI:** 10.1038/sj.bjc.6602376

**Published:** 2005-03-01

**Authors:** M Suzuki, C Hao, T Takahashi, H Shigematsu, N Shivapurkar, U G Sathyanarayana, T Iizasa, T Fujisawa, K Hiroshima, A F Gazdar

**Affiliations:** 1 Hamon Center for Therapeutic Oncology Research, Department of Pathology, University of Texas Southwestern Medical Center, Dallas, TX 75390, USA; 2 Department of Thoracic Surgery, Graduate School of Medicine, Chiba University, Chiba 260-8607, Japan; 3 Department of Basic Pathology, Graduate School of Medicine, Chiba University, Chiba 260-8607, Japan

**Keywords:** methylation, SPARC, lung cancer, immunostaining

## Abstract

*SPARC* (secreted protein acidic and rich in cysteine) is an extracellular Ca^2+^-binding matricellular glycoprotein associated with the regulation of cell adhesion and growth. We investigated loss of expression of *SPARC* gene and promoter methylation in lung cancers and correlated the data with clinicopathological features. We observed loss of *SPARC* expression in 12 of 20 (60%) lung cancer cell lines. Treatment of expression-negative cell lines with a demethylating agent restored expression in all cases. Methylation frequencies of *SPARC* gene were 55% in 20 lung cancer cell lines. Primary tumours had methylation at a rate of 69% (119 of 173), while nonmalignant lung tissues (*n*=60) had very low rates (3%). In lung adenocarcinomas, *SPARC* methylation correlated with a negative prognosis (*P*=0.0021; relative risk 4.65, 95% confidence interval 1.75–12.35, multivariate Cox's proportional-hazard model). Immunostaining revealed protein expression in bronchial epithelium (weak intensity) and in juxtatumoral stromal tissues (strong intensity) accompanied by frequent loss in cancer cells that correlated with the presence of methylation (*P*<0.001). Our findings are of biological interest and potentially of clinical importance in human lung cancers.

The matricellular protein SPARC (secreted protein acidic and rich in cysteine), also known as osteonectin/BM-40, is a calcium-binding glycoprotein that shows a high degree of interspecies sequence conservation and plays an important role in cell–matrix interactions during tissue remodelling, wound repair, morphogenesis, cellular differentiation, cell migration, and angiogenesis (Sage *et al*, 1989; Jendraschak and Sage, 1996; Yan and Sage, 1999; Bradshaw and Sage, 2001; Brekken and Sage, 2001). Its role in tumorigenesis is complex, and expression is often being downregulated in tumour cells accompanied by upregulation in juxtatumoral stromal cells. *SPARC* is highly expressed in reactive fibroblasts, and expression is deregulated in many types of human malignant tumours (Porte *et al*, 1995; Le Bail *et al*, 1999; Rempel *et al*, 1999; Paley *et al*, 2000). SPARC may promote vascularisation of tumours, tumour progression, or invasiveness by modulating the activity of cytokines and stimulating secretion of tissue remodelling metalloproteases (Lane and Sage, 1994; Motamed and Sage, 1997; Sage, 1997). Owing to the correlation between expression and invasion, SPARC was thought to be a proinvasive protein (Everitt and Sage, 1992a, 1992b; Lane *et al*, 1994; Ledda *et al*, 1997). However, ovarian cancer cells treated with SPARC showed inhibition of cell proliferation and underwent apoptosis (Yiu *et al*, 2001). SPARC potently inhibited angiogenesis and significantly impaired neuroblastoma tumour growth *in vivo* (Chlenski *et al*, 2002). Implanted Lewis lung carcinoma cells grew more rapidly in SPARC null mice (Brekken *et al*, 2003). Thus, the exact role of SPARC in tumour growth and progression is unclear.

The article "Aberrant methylation of SPARC in human lung cancers" was retracted in 2013. Reasons: misconduct by an author; duplicated data.

DNA methylation is a major mechanism associated with the inactivation of tumour suppressor genes in cancer (Esteller *et al*, 2001; Jones and Baylin, 2002; Suzuki *et al*, 2004). It has been reported that *SPARC* is silenced through DNA methylation in pancreatic cancer cells (Sato *et al*, 2003). SPARC protein by immunostaining was overexpressed in stromal fibroblasts immediately adjacent to the neoplastic epithelium in pancreatic cancers, suggesting SPARC expression in juxtatumoral tissues is regulated through tumour–stromal interactions (Sato *et al*, 2003). As exogenous SPARC inhibits the growth of pancreatic cancer cells *in vitro*, tumour–stromal interactions of SPARC may act to facilitate or retard tumour progression (Sato *et al*, 2003).

In non-small-cell lung cancer (NSCLC), SPARC expression by immunostaining was also found strongly in stromal fibroblasts, persistently in chondrocytes of bronchial cartilage, weakly in bronchial epithelium, but not in alveolar cells nor in tumour cells (Koukourakis *et al*, 2003). *SPARC*, is located at 5q33.1, a region that demonstrates frequent loss of heterozygosity in idiopathic pulmonary fibrosis and small-cell lung cancer (SCLC) (Girard *et al*, 2000; Demopoulos *et al*, 2002).

In this study, we examined the mRNA expression and methylation of *SPARC* in lung cancer cell lines, and examined the methylation and protein by immunostaining in primary tumours. We correlated these findings with clinicopathologic features.

## MATERIALS AND METHODS

### Cell lines and tumour samples

We studied 12 NSCLC cell lines (NCI-H460, NCI-H1437, NCI-H1770, NCI-H2087, NCI-H2122, NCI-H2126, HCC15, HCC95, HCC193, HCC366, HCC515, HCC1171) and eight SCLC cell lines (NCI-H69, NCI-H146, NCI-H209, NCI-H211, NCI-H524, NCI-H526, NCI-H1672, NCI-H2171) that were established by us (Phelps *et al*, 1996), several of which are deposited in the American Type Culture Collection (Manassas, VA, USA). Cell cultures were grown in RPMI-1640 medium (Life Technologies Inc., Rockville, MD, USA) supplemented with 5% fetal bovine serum and incubated in 5% CO_2_ at 37°C. Cell lines established at the National Cancer Institute have the prefix NCI, while those established at UT Southwestern Medical Center have the prefix HCC. Nonmalignant human bronchial epithelial cells (NHBEC) were cultured as reported previously (Toyooka *et al*, 2002), and normal trachea RNA was obtained from Clontech (Palo Alto, CA, USA).

The article "Aberrant methylation of SPARC in human lung cancers" was retracted in 2013. Reasons: misconduct by an author; duplicated data.

Surgically resected samples were obtained from patients with lung cancer who had not received treatment prior to resection at the Chiba University Hospital, Japan, after obtaining Institutional Review Board approval and informed consent. Samples were immediately frozen and stored at −80°C until used.

### Reverse transcription–polymerase chain reaction (RT–PCR) assay

An RT–PCR assay was used to examine *SPARC* mRNA expression. Total RNA was extracted from the samples with Trizol (Life Technologies, Rockville, MD, USA) following the manufacturer's instructions. RT reaction was performed on 4 *μ*g total RNA with deoxyribonuclease I and the SuperScript II First-Strand Synthesis using oligo-(dT) primer System (Life Technologies), and aliquots of the reaction mixture were used for the subsequent PCR amplification. The forward PCR amplification primer of *SPARC* was 5′-AAGATCCATGAGAATGAGAAG-3′ (Ex8-S), and the reverse primer 5′-AAAAGCGGGTGGTGCAATG-3′ (Ex9-AS) (Accession number NM_003118; forward, nucleotides 649–669; reverse, nucleotides 847–865). These sequences are separated by an intron, and we confirmed that genomic DNA was not amplified with these primers. Polymerase chain reaction amplification was carried out for 12 min at 95°C for initial denaturation, followed by 33 cycles of 94°C for 30 s, 60°C for 30 s, and 72°C for 45 s. The housekeeping gene *GAPDH* (glyceraldehyde-3-phosphate dehydrogenase) was used as an internal control to confirm the success of the RT reaction. The primers for *GAPDH* amplification were as follows: forward primer, 5′-CACTGGCGTCTTCACCACCATG-3′; and reverse primer, 5′-GCTTCACCACCTTCTTGATGTCA-3′. Polymerase chain reaction amplification was carried out for 12 min at 95°C for initial denaturation, followed by 25 cycles of 94°C for 30 s, 65°C for 45 s, and 72°C for 30 s. These primer sequences were identical to the human target genes as confirmed by a BLAST search. Polymerase chain reaction products were analysed on 2% agarose gels. Nonmalignant human bronchial and normal trachea were used as normal controls for RT–PCR.

The article "Aberrant methylation of SPARC in human lung cancers" was retracted in 2013. Reasons: misconduct by an author; duplicated data.

### 5-Aza-2′-deoxycytidine (5-Aza-CdR) treatment

In all, 11 tumour cell lines with *SPARC* hypermethylation and absent gene expression were incubated in culture medium with 4 *μ*M 5-Aza-CdR for 6 days, with medium changes on days 1, 3, and 5. The cells were harvested and RNA was extracted at day 6.

### DNA extraction and methylation-specific PCR (MSP)

Genomic DNA was obtained from cell lines, cultured nonmalignant cells, primary tumours, and nonmalignant tissues by digestion with proteinase K (Life Technologies), followed by phenol/chloroform (1 : 1) extraction (Herrmann and Frischauf, 1987). DNA methylation patterns in the CpG island of *SPARC* were determined by the method of MSP as reported by Herman *et al* (1996). Primer sequences of *SPARC* for unmethyalted reaction were 5′-TTTTTTAGATTGTTTGGAGAGTG-3′ (sense) and 5′-AACTAACAACATAAACAAAAATATC-3′ (antisense), and for the methylated reaction, 5′-GAGAGCGCGTTTTGTTTGTC-3′ (sense) and 5′-AACGACGTAAACGAAAATATCG-3′ (antisense) (Sato *et al*, 2003). Briefly, 1 *μ*g of genomic DNA was denatured by NaOH and modified by bisulfite. The modified DNA was purified using Wizard DNA purification kit (Promega, Madison, WI, USA), treated with NaOH to desulphonate, precipitated with ethanol, and resuspended in water. Polymerase chain reaction amplification was carried out for 12 min at 95°C for initial denaturation, followed by 38 cycles of 94°C for 20 s, 62°C for 20 s, and 72°C for 30 s. DNA from peripheral blood lymphocytes (*n*=14) from healthy nonsmoking subjects was used as negative controls for methylation-specific assays. DNA from lymphocytes of a healthy volunteer treated with *Sss*1 methyltransferase (New England BioLabs, Beverly, MA, USA) and then subjected to bisulfite treatment was used as a positive control for methylated alleles. Water blanks were included with each assay. Polymerase chain reaction products were visualised on 2% agarose gels stained with ethidium bromide.

### Immunostaining

SPARC was detected on paraffin-embedded tissue sections by the avidin–biotin peroxidase complex method using a mouse monoclonal antibody generated against the N-terminal region of SPARC (AON-5031; Hematologic Technologies Inc., Essex Junction, VT, USA). After immunostaining, the sections were counterstained with haematoxylin, dehydrated, and mounted.

Immunostaining was graded by two independent observers unaware of clinical or laboratory findings. Staining was categorised from 0 to 4+ based on the percentage of cells stained. Score 0 was assigned if less than 5% of cells were positive. A weak staining (+1) was assigned if 6–25% of cells were positive, a moderate staining (2+) was assigned if 26–50% of cells were positive, high sore (3+) was assigned if 51–75% of cells were positive, and a very high score (+4) was assigned if more than 75% of cells stained positive. The degree of staining intensity was also noted.

The article "Aberrant methylation of SPARC in human lung cancers" was retracted in 2013. Reasons: misconduct by an author; duplicated data.

### Statistical analysis

Statistical differences between groups were examined using Fisher's exact test, *χ*^2^ test, and Mann–Whitney test. Survival was calculated from the date of initial diagnosis until death or the date of the last follow-up (censored). Survival was analysed according to the Kaplan–Meier method, and differences in their distribution were evaluated by means of the log-rank test. A multivariate Cox's proportional-hazard model was developed to evaluate the covariates' joint effects. All *P*'s are two-sided, and *P* of less than 0.05 was defined as being statistically significant.

## RESULTS

### Aberrant methylation and expression of *SPARC* in cell lines

Expression of *SPARC* was examined by RT–PCR, and representative examples are shown in Figure 1A. *SPARC* expression was present in NHBEC and normal trachea. However, loss of *SPARC* expression was observed in 10 of 12 (83%) NSCLC cell lines, and two of eight (25%) SCLC cell lines (Table 1 and Figure 1B). Aberrant methylation was absent in DNA from peripheral blood lymphocytes from healthy nonsmoking volunteers (*n*=14) and NHBEC. Aberrant methylation was found in nine of 12 (75%) NSCLC cell lines, and two of eight (25%) SCLC cell lines. Both loss of expression and lack of methylation of *SPARC* were found in NSCLC cell line NCI-H2126, suggesting an alterative method of gene silencing in this cell line. The concordance between loss of gene expression and aberrant methylation of *SPARC* was 92% in NSCLC cell lines, and 100% in SCLC cell lines (overall concordance 95%).

### 5-Aza-2′-deoxycytidine treatment

Nine NSCLC cell lines (NCI-H460, NCI-H1437, NCI-H2087, NCI-H2122, HCC15, HCC95, HCC366, HCC515, HCC1171) and two SCLC cell lines (NCI-H146, NCI-H211) that showed loss of expression and methylation of *SPARC* were cultured with the demethylating agent 5-Aza-CdR. *SPARC* expression was restored after treatment in all 11 methylated cell lines tested (Figure 1C).

### Aberrant methylation of *SPARC* in primary tumours

Results of aberrant methylation of *SPARC* in primary tumours and nonmalignant tissues are detailed in Table 1 and Figure 1D. *SPARC* methylation was a tumour-specific event in lung cancers (*P*=0.0001) when compared with corresponding adjacent nonmalignant tissues.

Of 173 lung cancers, 119 (69%) were found to be methylated. There was a significant relationship between the major histologic types of lung cancer, NSCLC (115 of 161, 71%) and SCLC (four of 12, 33%) (*P*=0.01). When compared with clinicopathologic data, there was no significant association with gender, age, smoking history, or tumour stage. However, the frequency of methylation was significantly higher in squamous cell carcinomas (52 of 61, 85%) compared to adenocarcinomas (57 of 84, 68%) (*P*=0.01). Overall survival of adenocarcinomas was poorer in patients with *SPARC* methylation than in those without methylation (*P*=0.008; log-rank test; Figure 2) and for patients with advanced stages (*P*=0.0005). In a multivariate Cox's proportional-hazard model, promoter methylation of *SPARC* was an independent adverse prognostic factor (*P*=0.0021; relative risk (RR) 4.65, 95% confidence interval (CI) 1.75–12.35) next to stage (*P*=0.0003; RR 4.44, 95% CI 1.98–9.90) in adenocarcinoma cases (Table 2).

The article "Aberrant methylation of SPARC in human lung cancers" was retracted in 2013. Reasons: misconduct by an author; duplicated data.

### Immunostaining of SPARC protein in lung cancer

The expression of SPARC protein was examined in 162 primary lung cancers by immunostaining (Figure 3). In nonmalignant lung tissues, 73 of 128 cases (57%), negative (0) to weak (1+) SPARC expression was found in bronchial epithelial cell, while moderate (2+) to very strong (4+) expression was found in 55 cases. Alveolar cells were negative except for one case, which showed weak expression. Stromal fibroblasts distant from tumours showed negative to weak expression. Inflammatory cells including lymphocytes were negative expression, while chondrocytes of bronchial cartilage were moderate (2+) to strong (4+) SPARC expression. In 132 of 162 cases, negative (0) to weak (1+) SPARC expression was found in the cancer cells, while moderate (2+) to strong (4+) SPARC expression was found in 30 cases. Moderate (2+) to very strong (4+) SPARC expression was found in 154 of 162 cases in stromal cells near to or surrounding cancer cells. Thus, the predominant immunostaining pattern was negative in tumour cells while being positive in corresponding juxtatumoural stromal cells (125 of 162, 77%). However, there was no correlation of immunostaining pattern between tumour cells and stromal cells (Table 3A). Immunostaining pattern of neither tumour cells nor stromal cells correlated with patients' survival (data not shown). Of 162 cases, 105 showed loss (0) or weak (1+) expression of SPARC protein and methylation of *SPARC* gene, and 19 cases showed moderate (2+) to very strong (4+) expression without methylation (Table 3B). Thus, the concordance between methylation and loss of gene expression in tumour cells was 77% (*P*<0.0001). There was no correlation between tumour methylation and stromal cell immunostaining.

The article "Aberrant methylation of SPARC in human lung cancers" was retracted in 2013. Reasons: misconduct by an author; duplicated data.

## DISCUSSION

Sato *et al* demonstrated downregulation of *SPARC* mRNA in pancreatic cancer cells through DNA methylation (Sato *et al*, 2003). In our study, we observed that decreased *SPARC* expression in lung cancer cell lines is associated with DNA methylation of the gene promoter, and it is re-expressed by treatment with the demethylating agent 5-Aza-CdR in lung cancer cell lines. Although there are other possible mechanisms for downregulation of *SPARC* expression, the excellent concordance between mRNA expression by RT–PCR or protein expression by immunostaining and DNA methylation of *SPARC* indicates that the gene is downregulated mainly through DNA methylation in lung cancer.

As with other tumours, SPARC is downregulated in lung cancer cells while being upregulated in juxtatumoural stromal cells. Upregulation was unusual in stromal cells distant from the tumour. These findings result in a complex pattern of simultaneous selective downregulation in a specific cell type (tumour cells) accompanied by selective upregulation in adjacent stromal cells. A similar pattern has been previously described in ovarian, pancreatic, and lung cancers (Brown *et al*, 1999; Koukourakis *et al*, 2003; Sato *et al*, 2003). Our findings demonstrate that the mechanism of downregulation of SPARC in lung cancer cells is due to methylation. The dual up- and downregulation of SPARC in tumours makes interpretation difficult, while its role in tumorigenesis remains controversial. SPARC may function similar to TGF*β*, where signaling is downregulated in cancer cells early in tumorigenesis, but is overexpressed at later stages, thus acting either as tumour suppressor or oncogene, depending on the tumour stage (Wakefield and Roberts, 2002). Our data indicate that tumour–host interactions between lung cancer cells and stromal cells through SPARC protein play an important role in the pathogenesis of lung cancers.

Our data demonstrated that methylation of *SPARC* gene in tumour cells had poorer prognosis in lung adenocarcinomas, whereas reactivity of stromal fibroblasts had been reported to correlate worse prognosis in NSCLC (Koukourakis *et al*, 2003). The expression of SPARC in cancer tissues or functional analyses of *SPARC* gene in tumour cell lines have been widely studied (Table 4). Expression, as analysed by RT–PCR or immunostaining, was downregulated in lung, pancreatic, and ovarian cancers, whereas it was upregulated in oesophageal, bladder, metastatic prostate, hepatocellular cancers, and invasive meningiomas and malignant melanomas, and some of those findings were supported by functional analyses. The expression of SPARC by both normal and tumour cells is highly dependent on tumour type and culture conditions. Expression of SPARC in cancer tissues correlated with poor prognosis in malignant melanoma, bladder, and oesophageal carcinoma as also reported by others, although some of these reports was analysed by RT–PCR using whole specimens (Massi *et al*, 1999; Yamanaka *et al*, 2001; Yamashita *et al*, 2003). Aberrant expression of SPARC in primary tumours may result in negative prognosis.

The article "Aberrant methylation of SPARC in human lung cancers" was retracted in 2013. Reasons: misconduct by an author; duplicated data.

In conclusion, *SPARC* was downregulated in cancer cells through DNA methylation and overexpressed in its stromal cells of lung cancer, and DNA methylation correlated with prognosis in adenocarcinomas. DNA methylation of *SPARC* may play a role in the pathogenesis of lung cancers.

## Figures and Tables

**Figure 1:** (**A**) Representative examples of RT–PCR for *SPARC* in lung cancer cell lines, NHBEC, and normal trachea. *GAPDH* was used as a control for the RNA integrity and RT reactions. NC=negative control. (**B**) Representative examples of MSP assay in cell lines. Polymerase chain reaction products were visualised on 2% agarose gels stained with ethidium bromide. M=methylated band; U=unmethylated band. (**C**) Representative examples of RT–PCR for *SPARC* mRNA in lung cancer cell lines before (−) and after (+) treatment with 5-Aza-CdR. (**D**) Representative examples of MSP assay in primary tumours and nonmalignant tissues. All PCR products were visualised on 2% agarose gels stained with ethidium bromide. M=methylated band; U=unmethylated band; T=lung cancer tissues; N=nonmalignant lung tissue; PC=positive control.

**Figure 2:** Overall survival for 84 lung adenocarcinoma patients with early stages (*n*=34) or advanced stages (*n*=50) (**A**), or with (*n*=57) or without (*n*=27) the methylation of *SPARC* (**B**). Probability of survival curves was calculated using the Kaplan–Meier product-limit method and compared via the log-rank test between groups.

**Figure 3:** Immunostaining for SPARC in normal and malignant lung tissues. (**A**) Weak to moderate expression (1–2+) of SPARC by bronchial epithelium. Most of the staining is present in the apical surface of ciliated surface cells. (**B**) Bronchioli showed negative (0) expression. (**C**) Strong (3+) reactivity for SPARC in adenocarcinoma cells that lacked DNA methylation of *SPARC* gene, while alveolar cells and stromal cells are negative. (**D**) Negative immunostaining for SPARC in an adenocarcinoma demonstrating DNA methylation, while the adjacent stromal cells demonstrate very strong (4+) reactivity for SPARC; × 200 magnification.

**Table 1:** *SPARC* methylation in lung cancers

**Samples**	**Total no.**	**No. methylated (%)**
*Tumours*	193	
Cell lines		
NSCLC cell lines	12	9 (75)
SCLC cell lines	8	2 (25)
Primary NSCLC		
Adenocarcinoma	84	57 (68)
Squamous cell carcinoma	61	52 (85)
Large-cell carcinoma	11	6 (55)
Others	5	0 (0)
Primary SCLC	12	4 (33)
		
*Nonmalignant*	74	
Lung tissues and NHBEC	60	2 (3)
Peripheral blood mononuclear cells^a^	14	0 (0)

NSCLC=non-small-cell lung cancer; SCLC=small-cell lung cancer; NHBEC=nonmalignant human bronchial epithelial cells.

a From healthy nonsmoking volunteers.

The article "Aberrant methylation of SPARC in human lung cancers" was retracted in 2013. Reasons: misconduct by an author; duplicated data.

**Table 2:** Univariate and multivariate statistics of the prognostic value of gender, age, smoking, stage, and methylation status of *SPARC* for survival in lung adenocarcinomas

	**Number**	**Univariate** ***P*-value**	**Multivariate**		
			**Risk ratio**	**95% CI**	***P*-value**
*Gender*					
Female	40	0.76	0.71	0.30–1.65	0.42
Male	44				
					
*Age (years)*					
<64^a^	42	0.58	1.73	0.87–3.42	0.12
>64	42				
					
*Smoking*					
Nonsmoker	39	0.43	1.52	0.65–3.57	0.34
Smoker	45				
					
*Stage*					
I, II	34	0.0005	4.44	1.98–9.90	0.0003
III, IV	50				
					
*SPARC methylation*					
−	27	0.008	4.65	1.75–12.35	0.0021
+	57				

Results of univariate analyses using the log-rank test and multivariate analyses using Cox's proportional-hazard model of prognostic factors for overall survival. Stage and *SPARC* methylation are significantly associated with poor survival. CI=confidence interval; *SPARC*=secreted protein acidic and rich in cysteine.

a Divided by median age of adenocarcinoma cases.

**Table 3:** (A) SPARC immunostaining in tumour and stromal cell (*n*=162) and (B) methylation and immunostaining of SPARC in tumours (*n*=162)

**Tumour cell**	**Stromal cell**	**No. (%)**	***P*-value^a^**
*(A)*			
Positive	Positive^b^	29 (18)	>0.9
Positive	Negative^c^	1 (1)	
Negative	Positive	125 (77)	
Negative	Negative	7 (4)	
			

**Tumour methylation**	**Tumour immunostaining**	**No. (%)**	***P*-value**
*(B)*			
Methylated	Positive	11 (7)	<0.0001
Methylated	Negative	105 (65)	
Unmethylated	Positive	19 (12)	
Unmethylated	Negative	27 (17)	
			

**Tumour methylation**	**Stromal immunostaining**	**No. (%)**	***P*-value**
Methylated	Positive	110 (68)	>0.9
Methylated	Negative	6 (4)	
Unmethylated	Positive	44 (27)	
Unmethylated	Negative	2 (1)	

SPARC=secreted protein acidic and rich in cysteine.

a Fisher's exact probability.

b Positive reveals moderate (2+) to very strong (4+) immunostaining.

c Negative reveals negative (0) to weak (1+) immunostaining.

**Table 4:** (A) Expression of SPARC in various tumours and (B) functional analyses of SPARC for tumorigenesis in tumour cell lines

**Tumour type**	**Type of** **material**	**Method for detecting** **expression**	**Frequency or level of** **expression compared to** **nonmalignant tissues**	**Reference**
*(A)*				
Lung cancer	Tissue	RT–PCR	18%	Schneider *et al* (2004)
Lung cancer	Tissue	Immunostaining	5%	Koukourakis *et al* (2003)
Barrett's oesophagus	Tissue	RT–PCR	High (*P*=0.004)	Brabender *et al* (2003)
Pancreatic adenocarcinoma	Cell lines/tissue	RT–PCR/immunostaining	12%/32%	Sato *et al* (2003)
Oesopahgeal carcinoma	Tissue	Immunostaining	100%	Yamashita *et al* (2003)
Bladder cancer	Tissue	RT–PCR	High (*P*<0.0001)^a^	Yamanaka *et al* (2001)
Ovarian cancer	Tissue	Immunostaining	14%	Paley *et al* (2000)
Metastatic prostate cancer	Tissue	Immunostaining	High (most)^b^	Thomas *et al* (2000)
Invasive meningioma	Tissue	Immunostaining	100%	Rempel *et al* (1999)
Malignant melanoma	Tissue	Immunostaining	63.8%	Massi *et al* (1999)
Hepatocellular carcinoma	Tissue	Immunostaining	91%^c^	Le Bail *et al* (1999)
				

**Tumour type**	**Expression^d^**	**Effect for tumorigenesis**	**Reference**	
*(B)*				
Pancreatic adenocarcinoma	High	Growth suppression	Sato *et al* (2003)	
Prostate cancer	High	Promotion of cell migration to bone	De *et al* (2003)	
Lewis lung adenocarcinoma	Null	More rapid growth	Brekken *et al* (2003)	
Neuroblastoma	High	Impairing of tumour growth	Chlenski *et al* (2002)	
Breast cancer	High with c-Jun	Increase of motility and invasion	Briggs *et al* (2002)	
Glioma	High	Promotion of invasion	Schultz *et al* (2002)	
Ovarian cancer	High	Inhibition of the proliferation	Yiu *et al* (2001)	

SPARC=secreted protein acidic and rich in cysteine; RT–PCR=reverse transcription–polymerase chain reaction.

a Stage T2 or greater invasive tumours compared to stages T1 or less tumours.

b High levels of SPARC protein were observed in most of the metastatic foci.

c High in the stromal myofibroblasts of the tumour tissues.

d Forced expression by endogenous or exogenous SPARC.
